# Characteristics of Virulence Genes of Clinically Isolated Staphylococci in Jingzhou Area

**DOI:** 10.1155/2022/8804616

**Published:** 2022-07-30

**Authors:** Meng Wang, Qing Zhang

**Affiliations:** Yangtze University Health Science Center, Jingzhou 434020, China

## Abstract

**Purpose:**

The aim of this study was to further understand the distribution characteristics of staphylococcal virulence genes in the Jingzhou area, in order to provide a basis for clinically effective treatments and prevention and control measures.

**Methods:**

A total of 181 strains of staphylococci were collected from Jingzhou Hospital Affiliated to Yangtze University from April 2013 to April 2021, which were divided into the methicillin-resistant *Staphylococcus aureus* (MRSA) strains and the methicillin-sensitive *Staphylococcus aureus* (MSSA) strains and coagulase-negative staphylococci (CoNS) by an antimicrobial susceptibility test and PCR method. The 73 MRSA strains were classified by staphylococcal cassette chromosome mec (SCCmec) and *Staphylococcus* protein A (Spa). Sea, sec, seh, sek, seb, seq, sep, Tsst-1, clfA, clfB, fnbA, hla, hld, hlg, lukE, bbp, cna, eap, ebpS, sdrC, sdrD, sdrE, and Pvl genes were also detected in all strains. The *χ*^2^ test was used for statistical analysis for comparison between groups.

**Results:**

The 181 strains of staphylococci were divided into 97 strains of MRSA, 54 strains of MSSA, and 30 strains of CoNS. 73 MRSA strains were derived from clinical specimens such as lower respiratory tract, secretions, sepsis secreted by tissue infection, urine, and hydrothorax. There were 70 strains that can be identified including SCCmec types and 15 Spa types of all strains, while the most popular types were SCCmecIII-t030 and SCCmecIV-t437 from lower respiratory tract specimens. There were four virulence genes that were detected including seb, seq, clfB, and hld in CoNS strains, while the detection rates of these four virulence genes in *Staphylococcus aureus* were higher than that of CoNS, and the differences were statistically significant, *P* < 0.05(*P*=0.004, *P*=0.001, *P*=0.001, *P*=0.001). 23 virulence genes were detected in 151 strains of *Staphylococcus aureus*, among which the detection rate of the Tsst-1 gene was the lowest and that of the clfB gene was the highest, and the other genes were 4.6%∼98.0%. The detection rates of sea, sek, seb, seq, sep, cna, eap, ebpS, sdrC, and sdrE virulence genes in MRSA were higher than that of MSSA, and the differences were statistically significant, *P* < 0.05 (*P*=0.001, *P*=0.001, , *P*=0.001, *P*=0.001, *P*=0.009, , *P*=0.019, *P*=0.001, , *P*=0.001, *P*=0.001, , *P*=0.003).

**Conclusion:**

The mainly prevalent type of MRSA strains in Jingzhou is SCCmecIII-t030 in lower respiratory tract specimens. Virulence genes of *Staphylococcus aureus* and antibiotic drug resistance rates are also different from other regions. In this experiment, virulence genes were also detected in CoNS, suggesting that more attention should be paid to the prevention and treatment of these strains clinically.

## 1. Background

According to the monitoring data of the China Bacterial Resistance Surveillance Network in 2019, *Staphylococcus aureus* (*S. aureus*) accounted for 32.3% of Gram-positive bacteria, ranking first. Among them, the detection rate of methicillin-resistant *Staphylococcus aureus* (MRSA) showed a downward trend compared with last year, reflecting the potential threat of methicillin-susceptible *Staphylococcus aureus* (MSSA). In the meantime, the detection rate of methicillin-resistant MRSA in Hubei was 30.4% higher than the national average of 30.2% (http://www.carss.cn). *S. aureus* is an important Gram-positive pathogen which is one of the first pathogens to be studied. As one of the six “ESKAPE” organisms, it is a kind of opportunistic pathogen that can cause many types of infections in the human body with high toxicity. Because of multiple superantigen virulence genes, they have the threat of affecting the severity of patient infections and related complications and mortality, including blood, skin, soft tissue, and lower respiratory tract infections, toxin-mediated syndrome, and other life-threatening diseases, as well as infections related to medical devices, such as central-line associated bloodstream infection (CLABSI), and some seriously deep infections, such as endocarditis and osteomyelitis, and so on [1–3]. Due to the regional heterogeneity of the toxins expressed by the strains, this type of pathogen is potentially threatening in domestic and foreign hospital and community infections. In 1961, one year after methicillin was used in the clinical treatment of *S. aureus*, a type of bacteria, namely, methicillin-resistant *Staphylococcus aureus* (MRSA), was quickly isolated from the treated patients in clinic. Extensive drug resistance has made the treatment quite complicated, and a wide-ranging outbreak has occurred rapidly around the world, becoming one of the pathogens that still have a great threat in clinic [4]. *S. aureus* can secrete a variety of toxins and resist the normal defense of the host. The main *S. aureus* toxins can be divided into three categories: pore-forming toxins (PFTs), exfoliative toxins (ETs), and superantigens (SAgs), PFTs can be further divided into hemolysin, leukotoxin, and phenol soluble modulator protein (PSMs), and so on [5]. The adhesion of *S. aureus* to host epithelial cells is mediated by a type of cell wall-related proteins, which are named microbial surface components recognizing adhesive matrix molecules (MSCRAMMs) [6]; it is of great significance for the colonization of bacteria and the occurrence of invasive infections afterward. Infections caused by *S. aureus* are related to the formation of biofilms. The interaction of cell wall-anchored proteins (CWAPs) of bacteria plays an important role in the development of biofilms [7]. The classification of *S. aureus* virulence genes involved in the experiment is shown in Table 1. The type of *S. aureus* will not only change over time but also change differences in different regions. For example, the most prevalent staphylococcal protein A (Spa) types are t030 in Asia [8], t032 in Europe [9], t008 in America, t037 in Africa, and t020 in Australia [10]. In 2000, the domestic prevalent strain of *S. aureus* changed from t037-SCCmecIII to t030-SCCmecIII [11]. From 2013 to 2016, the domestic bacteremia caused by MRSA changed from t030-MRSA to t437-MRSA [12]. The most popular spa type in Hainan is t189, and the most common type of staphylococcal cassette chromosome mec (SCCmec) is SCCmecIV [13], t2460, and SCCmecII in Wuhan [2]. As of 2017, the spa type in Shanghai has gradually changed from t030 and t037 to t2460 [14]. Therefore, the purpose of this study is to understand the typing characteristics of MRSA strains prevalent in Jingzhou for the first time through experiments and to increase coagulase-negative staphylococci (CoNS) and MSSA strains to further understand the virulence genes of staphylococci in this region. The distribution type and epidemiological characteristics of the disease provide a theoretical basis for clinical prevention and control of epidemic spread, the establishment of effective measures, and clarification of pathogenic mechanisms.

## 2. Materials and Methods

### 2.1. Clinical Isolates

A total of 181 strains of staphylococci isolated from various clinical specimens of Jingzhou Hospital Affiliated to Yangtze University from April 2013 to April 2021 were collected. The staphylococci species were identified by a flight mass spectrometer (Microflex Brooke Dalton, Germany), and the mecA gene [15] was detected by a drug susceptibility test and PCR method (primer sequence was provided by Shenggong Biological Engineering Company, Shanghai, upstream: 5′-AGTTCTGCAGTACCGGATTTGC-3′, downstream: 5′-ATCGATGGTAAAGGTT GGC-3′), to confirm the strain type, and stored them at -80°C. A total of 97 strains of MRSA were derived from the lower respiratory tract (*n* = 67), secretions (*n* = 14), sepsis secreted by tissue infection (*n* = 10), urine (*n* = 3), and other samples (*n* = 3), including blood, pyoperitoneum, hydrothorax; a total of 54 strains of MSSA were derived from secretions (*n* = 15), blood (*n* = 12), sepsis secreted by tissue infection (*n* = 11), lower respiratory tract (*n* = 4), and other samples (*n* = 12), including ear swab, punctate, the tip of the catheter, joint fluid, urine, and drainage fluid; a total of 30 strains of CoNS were derived from the lower respiratory tract (*n* = 6), secretions (*n* = 6), blood (*n* = 6), urine (*n* = 4), and other samples (*n* = 8), including punctate, hydrothorax, cerebrospinal fluid (CSF), sepsis secreted by tissue infection. This study was approved by the Ethics Committee of Jingzhou Hospital Affiliated to Yangtze University.

### 2.2. Chromosomal DNA Extraction

We use lysozyme (A610308-0001, Shenggong Biological Engineering Company, Shanghai) and bacterial genomic DNA rapid extraction kit (B518225, Shenggong Biological Engineering Company, Shanghai) to extract DNA according to the instructions in the kit. The DNA mentioned is a template for PCR amplification.

### 2.3. SCCmec and Spa Typing

SCCmec and Spa typing were performed on 73 MRSA strains. We use primer sequences and molecular experimental methods in the literature described previously [16] to perform SCCmec typing and subtype detection of target strains. For the detection of Spa typing, first, the primer sequence in the PCR method was synthesized by Shenggong Biological Engineering Company, Shanghai, according to the report of Shopsin [17], upstream: 5′-TAAAGACGATCCTTCGGTGAGC-3′, downstream: 5′-CAGCAGTAGTGCCGTTTGCTT-3′. We use the amplification kit (TaKaRaTaq™(with Mg^2+^ free buffer), Takara Bio Inc., Japan) to operate through the instructions in it. The amplified products were electrophoresed on a 2% agarose gel, and the positive products obtained by the amplification were sequenced two-way by Shenggong Biological Engineering Company, Shanghai. The sequencing results were passed through the DNAGear software and the Spa typing database (http://www.ridom.de/spaserver) to determine the result of Spa typing of the target strain.

### 2.4. Detection of Virulence Genes

All 181 strains of staphylococci were tested for virulence genes. The upstream and downstream primer sequences of the virulence genes detected in this study were synthesized by Shenggong Biological Engineering Company, Shanghai. There are 23 virulence genes in total, and the primer sequences are from references [18–22]. We use the amplification kit (B532061, Shenggong Biological Engineering Company, Shanghai) according to the instructions in it. The amplified products were electrophoresed on a 1% agarose gel, and the gel imager took pictures to observe and record the results.

### 2.5. Antimicrobial Susceptibility Test (AST)

151 strains of *S. aureus* were tested for antimicrobial drug susceptibility (AST). AST used a VITEK 2 Compact system and the VITEK 2 AST-P639 Test Kit (bioMerieux, France) for testing. The VITEK 2 AST-P639 Test Kit contains 17 antibiotics: penicillin (PEN), oxacillin (OXA), cefoxitin (FOX), gentamicin (GEN), rifampicin (RIF), ciprofloxacin (CIP), levofloxacin (LVX), moxifloxacin (MFX), Bactrim (SXT), clindamycin (CLI), erythromycin (ERY), nitrofurantoin (NIT), linezolid (LNZ), vancomycin (VAN), quinupristin (QDA), tetracycline (TCY), and tigecycline (TGC). *S. aureus* ATCC29213 was used as the quality control strain for AST. The result analysis was based on the Clinical and Laboratory Standards Institute (CLSI) M100-S30 standard.

### 2.6. Statistical Analysis

The data were statistically analyzed using SPSS25.0 software, and the calculated data were expressed as a percentage. The comparison between groups was performed by the *χ*^2^ test, and *P* < 0.05 indicated that the difference was statistically significant.

## 3. Results

### 3.1. SCCmec and Spa Typing of MRSA

Among the 73 strains of MRSA, 70 strains could be clearly typed SCCmec, including SCCmecI (*n* = 2), SCCmecII (*n* = 1), SCCmecIII (*n* = 33), SCCmecIV (*n* = 26), and SCCmecV (*n* = 8). 52 strains came from the lower respiratory tract, 8 Spa types, mainly t030 (*n* = 29). 9 strains came from secretions, 5 Spa types, mainly t030 (*n* = 4). 9 strains came from sepsis secreted by tissue infection, 6 Spa types, mainly t437 (*n* = 3). The remaining 3 strains were from urine and hydrothorax, 2 Spa types, mainly t437 (*n* = 2). Based on the above results, the most common type of 73 MRSA strains were lower respiratory tract specimens SCCmecIII-t030 (*n* = 24) and SCCmecIV-t437 (*n* = 14). The results are presented in Table 2.

### 3.2. The Results of AST

*S. aureus* was sensitive to NIT, LNZ, VAN, and TGC and also highly sensitive to SXT (94%). Most strains were resistant to PEN (97.4%). The drug resistance rate to other antibiotics was between 30.5% and 68.2%. The drug resistance rates of MRSA were PEN (100%), GEN (49.5%), RIF (46.4%), CIP (54.6%), LVX (51.5%), MFX (49.5%), CLI (76.3%), ERY (80.4%), and TCY (66.7%). These results were higher than the results of MSSA, *P* < 0.05, and the differences were statistically significant. The drug resistance rates of MSSA were SXT (7.4%) and QDA (37.0%), which were higher than the results of MRSA, *P* > 0.05, and the differences were not statistically significant. The results are presented in Table 3.

MRSA with Spa type t030 and t437 were sensitive to NIT, LNZ, VAN, and TGC and also highly sensitive to SXT (98.2%). All strains were resistant to PEN. The drug resistance rate to other antibiotics was between 36.8% and 84.2%. The drug resistance rates of t030 were GEN (100.0%), RIF (100.0%), CIP (100.0%), LVX (100.0%), MFX (100.0%), QDA (57.1%), and TCY (97.1%). These results were higher than the results of t437, *P* < 0.05, and the differences were statistically significant. The drug resistance rates of t437 were SXT (4.5%), CLI (90.9%), and ERY (95.5%), which were higher than the results of t030, *P* > 0.05, and the differences were not statistically significant. The results are presented in Table 4.

### 3.3. The Results of Virulence Genes

All virulence genes were detected in 181 strains of staphylococci. Among them, the results of Tsst-1 and sep genes were 2.2% and 3.9%. The result of clfB gene was 89.0%, while clfA and hla genes were followed by 81.8%, and the other virulence genes detection rate was between 6.1% and 80.7%. Four virulence genes, seb, seq, clfB, and hld, were detected in the strains of CoNS. The result of clfB gene was 40.0%, and the results of seb and hld genes were 3.3%. Statistical analysis showed that the results of these four virulence genes in *S. aureus* were higher than that of CoNS, and the differences were statistically significant, *P* < 0.05. The results are presented in Table 5.

All virulence genes were detected in 151 strains of *S. aureus*. Among them, the results of Tsst-1 and sep genes were 2.7% and 4.6%. The result of the clfB gene was 98.7%, while clfA and hla genes were followed by 98.0%, and the other virulence genes detection rate was between 7.3% and 96.7%. The result of sep gene in MRSA was 1.0%, while the results of clfB, clfA, hla, and other virulence genes were 97.9%, and the detection rate of other virulence genes was between 3.1% and 96.9%. As for MSSA, the results of seh and Tsst-1 genes were low at 1.9%, and the result of clfB gene was high at 100.0%, and the detection rate of the other virulence genes was between 3.7% and 98.2%. Statistical analysis showed that the results of virulence genes such as sea, sek, seb, seq, sep, cna, eap, ebpS, sdrC, and sdrE in MRSA were higher than that of MSSA, and the differences were statistically significant, *P* < 0.05. The results of virulence genes such as sec, seh, Tsst-1, fnbA, and hlg in MRSA were higher than that of MSSA, and the differences were not statistically significant, *P* > 0.05, while the results of virulence genes such as clfA, clfB, hla, hld, lukE, bbp, sdrD, and Pvl in MSSA were higher than those of MRSA, and the differences were not statistically significant, *P* > 0.05. The results are presented in Table 6.

Except for the sep and Tsst-1 genes that were not detected, the remaining virulence genes were detected in MRSA with Spa type t030 and t437. Among them, the results of virulence genes such as clfA, clfB, fnbA, hla, hlg, bbp, ebpS, and sdrE were high at 100.0%, and the sec gene was low at 1.8%. The results of remaining virulence genes were between 8.8% and 93.0%. The result of the sec gene in t030 was 2.9%, while the results of cna, lukE, and sdrD were 100%, and the results of other genes were between 5.7% and 97.1%. The sec and sdrC genes in t437 were not detected, while the result of the hld gene was 100%, and the results of other genes were between 4.6% and 90.9%. Statistical analysis showed that the results of virulence genes such as sea, lukE, cna, eap, sdrC, and sdrD in t030 were higher than those of t437, and the differences were statistically significant, *P* < 0.05. The result of the sec gene in t030 was higher than that of t437, and the difference was not statistically significant, *P* > 0.05. The results of virulence genes in t437 such as sek, seb, and Pvl were higher than those of t030, and the differences were statistically significant, *P* < 0.05. The results of virulence genes in t437 such as seh, seq, and hld were higher than those of t030, and the differences were not statistically significant, *P* > 0.05. The results are presented in Table 7.

## 4. Discussion

*S. aureus* is one of the human normal flora, and the main colonization sites are the skin and vestibule, while its asymptomatic colonization is about 30% in the nasal cavity of healthy adults [23]. Because it carries a variety of virulence genes, the prevention of its invasiveness and infection is particularly important. Relevant literature [5] shows that toxins can cause a weak host response, degrade cell-to-cell connections, and manipulate the immune response, which significantly contributes to the proliferation of *S. aureus*. Cell wall-related proteins can increase the colonization of *S. aureus* in the host and cause invasive infections. In addition, the typing method can increase the awareness of the epidemic types of strains and compare with other regions to understand the development and evolution trend of strains in this region.

The SCCmec and Spa typing of MRSA reflect the popular clones of strains in different regions. Our study found that SCCmecIII was the most, which was consistent with the results of Guangdong [1] and Xinjiang [24], but different from those of Wuhan [2], Hainan [13], Shanghai [14], Beijing [25], where the most SCCmec types were SCCmecII and SCCmecIV, but SCCmecII was the least among our study. From the related literature [10], we found that Spa typing has different popular types all over the world. The most popular Spa typing in Asia are t030, t037, and t002, and those in Europe are t032, t008, and t002, while those in the United States are t008, t002, and t242, and those in Africa are t037, t84, and t064, while those in Australia are t202, t037, and t437. The main Spa typing in our study was t030, which was consistent with the above research's results, but different from those of Wuhan [2], Shanghai [14], Hainan [13], and Beijing [25], in which the main Spa types were t2460, t116 and t437. It shows the characteristics of the epidemic types of MRSA in Jingzhou. At the same time, understanding the epidemic types of strains in different regions also reflects the different evolutionary of strains. It can be used as a powerful reference for clinical medication and prevention in different regions.

In the results of AST, the results of *S. aureus* in RIF, GEN, LVX, CLI, ERY, and PEN were 30.5%, 33.1%, 34.4%, 63.6%, 68.2%, and 97.4% higher than the average resistance rates of *S. aureus* in the 2019 (http://www.carss.cn), which were 3.2%, 12.4%, 14.5%, 34.8%, 59.9%, and 92.5%. VAN and LNZ were both sensitive, and our results for SXT were 6.0%, which was lower than the average resistance rate, 13.6%. In addition, according to the results of the antimicrobial resistance website (http://www.chinets.com) until September 2021, the average drug resistance rates of MRSA in RIF, GEN, CIP, LVX, CLI, and ERY were 5.7%, 19.0%, 30.9%, 32.3%, 57.8%, and 74.9%, which were lower than the results of MRSA in our study, 46.4%, 49.5%, 54.6%, 51.5%, 76.3%, and 80.4%, while the results of VAN, LNZ, and PEN were consistent of 0 and 100.0%. The results of SXT and TGC were 5.2% and 0 which were lower than the average resistance rates, 7.5% and 0.7%. The average resistance rates of MSSA in RIF, CLI, ERY, and PEN were 0.9%, 17.9%, 46.2%, and 87.6% which were lower than the results of MSSA in our study, 1.9%, 40.7%, 46.3%, and 92.6%. VAN and LNZ were both sensitive. Our results of TGC, SXT, GEN, CIP, and LVX were 0, 7.4%, 3.7%, 3.7%, and 3.7%, which were lower than the average drug resistance rate, 0.1%, 14.2%, 7.7%, 11.4%, and 10.8%. Combining the analysis of the above results, we can find the uniqueness of the drug resistance rate of *S. aureus* in the Jingzhou area, which can be used as a reference for clinical medication. In addition, in our results, the results of MRSA were higher than that of MSSA, and the differences were statistically significant, *P* < 0.05. Due to the large number of MRSA with Spa type t030 and t437 in the typing results, in order to understand the drug resistance rates of the two types, we also conducted a drug sensitivity analysis. They were both sensitive to NIT, LNZ, VAN, and TGC, and we also found that the t030 was sensitive to SXT but had a high resistance rate to other antibiotics between 57.1% and 100.0%, which was basically higher than that of the t437, and the differences were statistically significant, *P* < 0.05. This may be the reason why the t030 is more popular in the Jingzhou area. It should attract more clinical attention.

The existence of virulence genes is one of the main reasons why *S. aureus* causes different clinical manifestations in patients, leading to epidemic infections in hospitals and communities [26]. Literature [5, 27, 28] show that hla can cause the lysis of erythrocyte, platelets, endothelial cells, epithelial cells, and some leukocyte; Pvl and hlg are specific, targeting human and rabbits leukocyte, the latter also includes human erythrocyte and neutrophils; lukE endows toxins with extensive leukocidal activity and is an important virulence gene of *S. aureus*; vomiting and diarrhea are one of the key characteristics of staphylococci food poisoning, and the protein disulfide are expressed by enterotoxin genes ring-related; Tsst-1 can cause toxic shock syndrome (TSS), involving multiple systems and organs of the human body; hld is a part of the core genome that encodes PSMs. Eap is an immune escape protein that plays a key role in the pathogenesis and survival of *S. aureus* [29]. The results of virulence genes in MRSA in our study were consistent with the results of 136 strains of MRSA reported by Li et al. [30]. On this basis, our study also added the detection of virulence genes in the MSSA and the CoNS to expand the research to understand the distribution of virulence genes among clinically isolated staphylococci in the Jingzhou area. Four virulence genes, mainly clfB (40.0%), were detected in the CoNS. The result of clfB (98.7%) in *S. aureus* was also the highest, which was different from other regions in China, mainly clfA and hla [13, 31, 32]. The results reflected the regional differences in the prevalence of virulence genes and suggested that certain preventive measures should also be taken for CoNS. In our study, the main MSCRAMMs of *S. aureus* were clfB (98.7%), clfA and hla (98.0%), hlg (96.7%), but sdrC (37.1%) was the lowest. The results of MRSA were generally higher than that of MSSA. Among them, the results between the two groups of 13 genes including sec, seh, Tsst-1, clfA, clfB, fnbA, hla, hld, hlg, lukE, bbp, sdrD, and Pvl. The differences were not statistically significant, *P* > 0.05. In addition, the statistical results of the detection rate of virulence genes between MRSA and MSSA were basically the same as the results of the study by Geng et al. [25], and the results of Pvl and sea genes in MRSA were 13.4% and 49.5% which were consistent with the findings of Fu et al. The authors of [2] reported that the results of the two genes in 131 MRSA were 10.7% and 48.1%, but the results of sec and seh genes were 54.2% and 18.3%, which were higher than our study, 14.4% and 10.3%. The results of eap and sdrC in 136 MRSA reported by Shipeng Li et al. [30] were 70.6% and 99.3%, which were higher than our study, 57.7% and 48.5%, but cna and sdrD were both 41.2%, which were lower than our study, 74.2% and 55.7%. The reasons for the different results may be the genetic factors of the strains, the regional environment, the different sources of specimens, and other factors, reflecting the necessity of further systematic research. In addition, our research also added the analysis of virulence genes carried by MRSA strains of Spa type t030 and t437. The results showed that, except for sep, Tsst-1 which were not detected by the two types, the results of clfA, clfB, fnbA, hla, hlg, bbp, ebpS, and sdrE were 100%, and the results of t030 are higher than that of t437, and the differences were statistically significant, *P* < 0.05. Combined with the AST results, it further reflected the reason why MRSA with Spa type t030 was more popular in the Jingzhou area which suggested that this type was clinically dangerous, and certain preventive measures should be taken.

In summary, the link between different toxins in *S. aureus* and certain specific disease symptoms has been established, such as enterotoxin, hemolysin, leukocidin, and toxic shock syndrome toxins. The interaction between secreted proteins and cell wall-related proteins facilitates the colonization and spread of bacteria and the formation of immune evasion. Therefore, understanding the distribution of virulence genes is of great significance for clinical prevention and treatment. At the same time, virulence genes were also detected in the CoNS in this experiment, suggesting the potential danger of this type. In addition, in terms of virulence genes, molecular typing, and antibiotic resistance rates, the results of the Jingzhou area are unique. Especially in the analysis of the MRSA with Spa type t030, the results of the drug resistance rate and virulence genes were high, which reflected the important significance of this research. Therefore, a further understanding of the epidemiological characteristics of staphylococci virulence genes in this region has a certain warning effect for effective clinical control measures.

## Figures and Tables

**Table 1:** Classification of *S. aureus* virulence genes.

PFTs			SAgs	Cell wall-related proteins and factors
Hemolysin	Leukotoxin	PSMs		
Hla	Pvl, lukE, hlg	hld	sea, sec, seh, sek, seb, seq sep, Tsst-1	fnbA, clfA, clfB, eap, sdrC, sdrD, sdrE

**Table 2:** Molecular types of different samples of MRSA.

Specimen sources	Spa types	SCCmec types	Quantity (*n*)
Lower respiratory tract	t030	III	24
		V	5
	t114	IV	1
	t116	IV	2
	t14314	IV	1
	t189	—	1
	t437	I	1
		IV	14
	t632	III	2
	t664	IV	1

Secretions	t030	III	4
	t1685	—	1
	t437	IV	1
		V	1
	t543	V	1
	t8886	IV	1

Sepsis	t030	III	2
	t078	—	1
	t114	IV	1
	t233	III	1
	t437	IV	2
		V	1
	t899	I	1

Urine	t311	II	1
	t437	IV	1

Hydrothorax	t437	IV	1

*Note*. “—” indicates that the classification was not clear.

**Table 3:** The distribution of antimicrobial resistance of MRSA and MSSA (%).

Antibiotics	Total strains (*n* = 151)	MRSA (*n* = 97)	MSSA (*n* = 54)	*χ* ^2^	*P*
PEN	147 (97.4)	97 (100.0)	50 (92.6)	—	0.015
OXA	97 (64.2)	97 (100.0)	0	151.000	0.001
FOX	97 (64.2)	97 (100.0)	0	151.000	0.001
GEN	50 (33.1)	48 (49.5)	2 (3.7)	32.826	0.001
RIF	46 (30.5)	45 (46.4)	1 (1.9)	32.486	0.001
CIP	55 (36.4)	53 (54.6)	2 (3.7)	38.864	0.001
LVX	52 (34.4)	50 (51.5)	2 (3.7)	35.167	0.001
MFX	50 (33.1)	48 (49.5)	2 (3.7)	32.826	0.001
SXT	9 (6.0)	5 (5.2)	4 (7.4)	0.041	0.840
CLI	96 (63.6)	74 (76.3)	22 (40.7)	18.929	0.001
ERY	103 (68.2)	78 (80.4)	25 (46.3)	18.620	0.001
NIT	0	0	0		
LNZ	0	0	0		
VAN	0	0	0		
QDA	52 (34.4)	32 (33.3)	20 (37.0)	0.252	0.616
TCY	72 (47.7)	65 (66.7)	7 (13.0)	40.619	0.001
TGC	0	0	0		

*Note*. “—” indicates the result of using Fisher's exact probability test.

**Table 4:** The distribution of antimicrobial resistance of t030 and t437 in MRSA (%).

Antibiotics	Total strains (*n* = 57)	t030 (*n* = 35)	t437 (*n* = 22)	*χ* ^2^	*P*
PEN	57 (100.0)	35 (100.0)	22 (100.0)		
OXA	57 (100.0)	35 (100.0)	22 (100.0)		
FOX	57 (100.0)	35 (100.0)	22 (100.0)		
GEN	37 (64.9)	35 (100.0)	2 (9.1)	49.017	0.001
RIF	36 (63.2)	35 (100.0)	1 (4.5)	52.898	0.001
CIP	36 (63.2)	35 (100.0)	1 (4.5)	52.898	0.001
LVX	36 (63.2)	35 (100.0)	1 (4.5)	52.898	0.001
MFX	36 (63.2)	35 (100.0)	1 (4.5)	52.898	0.001
SXT	1 (1.8)	0	1 (4.5)	—	0.386
CLI	46 (80.7)	26 (74.3)	20 (90.9)	1.448	0.229
ERY	48 (84.2)	27 (77.1)	21 (95.5)	2.169	0.141
NIT	0	0	0		
LNZ	0	0	0		
VAN	0	0	0		
QDA	21 (36.8)	20 (57.1)	1 (4.5)	16.061	0.001
TCY	46 (80.7)	34 (97.1)	12 (54.5)	13.123	0.001
TGC	0	0	0		

*Note*. “—” indicates the result of using Fisher's exact probability test.

**Table 5:** The distribution of virulence genes of 181 strains of *Staphylococci* (%).

Virulence genes	Total strains (*n* = 181)	*S. aureus* (*n* = 151)	CoNS (*n* = 30)	*χ* ^2^	*P*
sea	55 (30.4)	55 (36.4)	—		
sec	19 (10.5)	19 (12.6)	—		
seh	11 (6.1)	11 (7.3)	—		
sek	38 (21.0)	38 (25.2)	—		
seb	43 (23.8)	42 (27.8)	1 (3.3)	8.281	0.004
seq	101 (55.8)	96 (63.6)	5 (16.7)	22.330	0.001
sep	7 (3.9)	7 (4.6)	—		
Tsst-1	4 (2.2)	4 (2.7)	—		
clfA	148 (81.8)	148 (98.0)	—		
clfB	161 (89.0)	149 (98.7)	12 (40.0)	81.799	0.001
fnbA	144 (79.6)	144 (95.4)	—		
hla	148 (81.8)	148 (98.0)	—		
hld	144 (79.6)	143 (94.7)	1 (3.3)	128.472	0.001
hlg	146 (80.7)	146 (96.7)	—		
lukE	96 (53.0)	96 (63.6)	—		
bbp	137 (75.7)	137 (90.7)	—		
cna	102 (56.4)	102 (67.6)	—		
eap	67 (37.0)	67 (44.4)	—		
ebpS	137 (75.7)	137 (90.7)	—		
sdrC	56 (30.9)	56 (37.1)	—		
sdrD	87 (48.1)	87 (57.6)	—		
sdrE	125 (69.1)	125 (82.8)	—		
Pvl	23 (12.7)	23 (15.2)	—		

*Note*. “—” indicates that was not detected.

**Table 6:** The distribution of virulence genes of 151 strains of *S. aureus* (%).

Virulence genes	Total strains (*n* = 151)	MRSA (*n* = 97)	MSSA (*n* = 54)	*χ* ^2^	*P*
sea	55 (36.4)	48 (49.5)	7 (13.0)	19.981	0.001
sec	19 (12.6)	14 (14.4)	5 (9.3)	0.844	0.358
seh	11 (7.3)	10 (10.3)	1 (1.9)	2.528	0.112
sek	38 (25.2)	36 (37.1)	2 (3.7)	20.560	0.001
seb	42 (27.8)	37 (38.1)	5 (9.3)	14.415	0.001
seq	96 (63.6)	84 (86.6)	12 (22.2)	62.080	0.001
sep	7 (4.6)	1 (1.0)	6 (11.1)	—	0.009
Tsst-1	4 (2.7)	3 (3.1)	1 (1.9)	—	1.000
clfA	148 (98.0)	95 (97.9)	53 (98.2)	—	1.000
clfB	149 (98.7)	95 (97.9)	54 (100.0)	—	0.537
fnbA	144 (95.4)	94 (96.9)	50 (92.6)	—	0.249
hla	148 (98.0)	95 (97.9)	53 (98.2)	—	1.000
hld	143 (94.7)	90 (92.8)	53 (98.2)	1.064	0.302
hlg	146 (96.7)	94 (96.9)	52 (96.3)	—	1.000
lukE	96 (63.6)	59 (60.8)	37 (68.5)	0.887	0.346
bbp	137 (90.7)	87 (89.7)	50 (92.6)	0.347	0.556
cna	102 (67.6)	72 (74.2)	30 (55.6)	5.517	0.019
eap	67 (44.4)	56 (57.7)	11 (20.4)	19.617	0.001
ebpS	137 (90.7)	94 (96.9)	43 (79.6)	12.310	0.001
sdrC	56 (37.1)	47 (48.5)	9 (16.7)	15.022	0.001
sdrD	87 (57.6)	54 (55.7)	33 (61.1)	0.421	0.517
sdrE	125 (82.8)	87 (89.7)	38 (70.4)	9.084	0.003
Pvl	23 (15.2)	13 (13.4)	10 (18.5)	0.703	0.402

*Note*. “—” indicates the result of using Fisher's exact probability test.

**Table 7:** The distribution of virulence genes of t030 and t437 in MRSA (%).

Virulence genes	Total strain (*n* = 57)	t030 (*n* = 35)	t437 (*n* = 22)	*χ* ^2^	*P*
sea	38 (66.7)	34 (97.1)	4 (18.2)	37.901	0.001
sec	1 (1.8)	1 (2.9)	0	—	1.000
seh	5 (8.8)	3 (8.6)	2 (9.1)	—	1.000
sek	24 (42.1)	6 (17.1)	18 (81.8)	23.180	0.001
seb	23 (40.4)	3 (8.6)	20 (90.9)	38.050	0.001
seq	50 (87.7)	30 (85.7)	20 (90.9)	—	0.695
sep	0	0	0		
Tsst-1	0	0	0		
clfa	57 (100.0)	35 (100.0)	22 (100.0)		
clfb	57 (100.0)	35 (100.0)	22 (100.0)		
fnba	57 (100.0)	35 (100.0)	22 (100.0)		
hla	57 (100.0)	35 (100.0)	22 (100.0)		
hld	53 (93.0)	31 (88.6)	22 (100.0)	—	0.151
hlg	57 (100.0)	35 (100.0)	22 (100.0)		
luke	38 (66.7)	35 (100.0)	3 (13.6)	45.341	0.001
bbp	57 (100.0)	35 (100.0)	22 (100.0)		
cna	44 (77.2)	35 (100.0)	9 (40.9)	26.792	0.001
eap	40 (70.2)	34 (97.1)	6 (27.3)	31.509	0.001
ebps	57 (100.0)	35 (100.0)	22 (100.0)		
sdrc	34 (59.7)	34 (97.1)	0	52.964	0.001
sdrd	36 (63.2)	35 (100.0)	1 (4.6)	52.898	0.001
sdre	57 (100.0)	35 (100.0)	22 (100.0)		
Pvl	10 (17.5)	2 (5.7)	8 (36.4)	6.781	0.009

*Note*. “—” indicates the result of using Fisher's exact probability test.

## Data Availability

The data used to support the findings of this study are available from the corresponding author upon request.
